# HMGB1 Facilitated Macrophage Reprogramming towards a Proinflammatory M1-like Phenotype in Experimental Autoimmune Myocarditis Development

**DOI:** 10.1038/srep21884

**Published:** 2016-02-22

**Authors:** Zhaoliang Su, Pan Zhang, Ying Yu, Hongxiang Lu, Yanfang Liu, Ping Ni, Xiaolian Su, Dan Wang, Yueqin Liu, Jia Wang, Huiling Shen, Wenlin Xu, Huaxi Xu

**Affiliations:** 1 Department of Immunology, Jiangsu University, Zhenjiang, China, 212013; 2 The Central Laboratory, the Fourth Affiliated Hospital of Jiangsu University, Zhenjiang, China, 212001

## Abstract

Macrophages can be reprogramming, such as the classical activated macrophage, M1 or alternative activated macrophages, M2 phenotype following the milieu danger signals, especially inflammatory factors. Macrophage reprogramming is now considered as a key determinant of disease development and/or regression. Experimental autoimmune myocarditis (EAM) is characterized by monocytes/macrophage infiltration, Th17 cells activation and inflammatory factors producing such as high mobility group box 1 (HMGB1). Whether infiltrated macrophages could be reprogramming in EAM? HMGB1 was associated with macrophage reprogramming? Our results clearly demonstrated that infiltrated macrophage was reprogrammed towards a proinflammatory M1-like phenotype and cardiac protection by monocytes/macrophages depletion or HMGB1 blockade in EAM; *in vitro*, HMGB1 facilitated macrophage reprogramming towards M1-like phenotype dependent on TLR4-PI3Kγ-Erk1/2 pathway; furthermore, the reprogramming M1-like macrophage promoted Th17 expansion. Therefore, we speculated that HMGB1 contributed EAM development via facilitating macrophage reprogramming towards M1-like phenotype except for directly modulating Th17 cells expansion.

Macrophages, as highly plastic cells, play critical roles in autoimmune diseases, cancers and inflammatory diseases^1^,^2^. Macrophages can reprogram their phenotype toward proinflammatory M1 phenotype or anti-inflammatory M2 phenotype^2^,^3^,^4^. M1 macrophage produces various proinflammatory cytokines, such as IL-6, IL-1β, TNF-α, monocyte chemoattractant protein-1 (MCP-1) and up-regulate MHCII, CD86/CD80. Conversely, M2 macrophage preferentially secretes high levels of anti-inflammatory cytokines, such as IL-10, increases Arg-1 activity, up-regulated macrophage mannose receptor (MMR) expression, involves in the anti-inflammatory and remodeling^5^,^6^. Recent data indicates that macrophage can reprogram their functional phenotype following the different inflammatory microenvironment^7^,^8^.

High mobility group box 1 (HMGB1), as an important inflammatory factor or an alarmin, not only was involved in the response to infection, but also associate with cell differentiation, migration, tumor metastasis and many autoimmune diseases^9^,^10^,^11^. Our previous data has shown HMGB1 was significantly up-regulation both in heart tissue and blood in experimental autoimmune myocarditis (EAM). EAM, a CD4^+^ Th17 cell mediated inflammatory diseases, is characterized by lots of monocytes/macrophages infiltration, cardiac myocytes’ necrosis, cardiac fibroblasts’ proliferation, collagen deposition and myocardial fibrosis^12^,^13^,^14^. And our results also showed that HMGB1 blockade attenuated cardiac pathological changes via directly modulating Th17 cells expansion, decreased monocytes/macrophages infiltration and collagen deposition^13^. However, no any data indicated whether HMGB1 up-regulation was associated with macrophage reprogramming?

Therefore, the present work was to address whether HMGB1 could contribute to EAM development via facilitating infiltrated macrophages reprogramming?Our results clearly demonstrated that infiltrated macrophage was reprogrammed towards a proinflammatory M1-like phenotype and cardiac protection by monocytes/macrophages depletion or HMGB1 blockade in EAM; *in vitro*, HMGB1 facilitated macrophage reprogramming towards M1-like phenotype dependent on TLR4-PI3Kγ-Erk1/2 pathway; and reprogramming M1-like macrophage promoted Th17 cells expansion.

## Results

### M1-like macrophage was infiltration in heart tissue and cardiac protection by monocytes/macrophages depletion in EAM

Our previous data showed that Th17 cells mediated the EAM development and monocytes/macrophages infiltrated the heart^13^,^14^. And the phenotype of macrophages infiltrated in heart was determined. As Fig. 1A showed that F4/80^+^CD11C^+^macrophages were predominant in EAM (15 folds comparing with control, *p* < 0.001). To furthering confirm the infiltrated macrophages involving in EAM development. The monocytes/macrophages were deleted by clodronate liposome before the EAM induction. The monocytes/macrophages depletion results in a reduction of Th17 cells infiltration and cardiac protection; the gross severity scores were obviously lower than EAM group (2.2 ± 0.84 vs 4.6 ± 0.55, respectively, *p* < 0.001, Fig. 1B); IL-6, IL-1β and TNF-α were also obviously decreased comparing with EAM group (IL-6: 139.20 ± 69.61 pg/mL vs 374.24 ± 115.03 pg/mL, *p* < 0.001; IL-1β: 13.34 ± 5.88 pg/mL vs 26.78 ± 17.82 pg/mL, *p* < 0.05; and TNF-α: 183.20 ± 25.34 pg/mL vs 381.80 ± 66.14 pg/mL, *p* < 0.001; respectively) and the control groups were 15.3 ± 7.67 pg/mL, 7.20 ± 0.57 pg/mL and 26.20 ± 8.26 pg/mL, respectively (Fig. 1C). Taken together, these results demonstrate that M1-like macrophage infiltration was predominant and cardiac protection by monocytes/macrophages depletion in EAM.

### HMGB1 Facilitated Macrophage Reprogramming towards a Proinflammatory M1-like Phenotype *in vitro*

And then next question was whether HMGB1 was associated with macrophage reprogramming towards a M1-like phenotype. Therefore, ANA-1 macrophages and peritoneal macrophages were incubated with 100 ng/ml recombinant HMGB1, 500 ng/ml LPS or without, respectively. After 12 h, iNOS expression was obviously increased, conversely, the Arg-1 expression was decreased (Fig. 2B, *p* < 0.05); however, the iNOS increasing was not a dose-dependent manner (Fig. 2A); the western blot data was furthering confirm it (Fig. 2C). The iNOS activities detection was also demonstrated that iNOS expression was up-regulated (Fig. 2D).

The M1 macrophage associated cytokines, IL-6, TNF-α, IL-1α, IL-1β and MCP-1 mRNA expression were obviously increased (9.7 folds, 20 folds, 7.7 folds, 11.3 fold and 22 folds vs controls, respectively, *p* < 0.001, Fig. 2E). And double staining with F4/80 and CD11c antibodies furthering indicated that HMGB1 increased CD11c^+^F4/80^+^macrophages comparing with BSA group (56.78 ± 8.02% vs 5.02 ± 2.93%, *p* < 0.05); after TLR4 blockade on macrophages by mAb, the proportion of CD11c^+^F4/80^+^macrophages was decreased following HMGB1 treatment (18.00 ± 5.74%) (Fig. 2F). Additionally, HMGB1 could also promote the ANA-1 migration (Fig. 2G). Furthermore, M1-like macrophages preferentially expressed HMGB1 (Supplementary Figure 1). Taken together, these results clearly demonstrate that HMGB1 facilitated macrophage reprogramming towards a proinflammatory M1-like phenotype via ligation with TLR4 *in vitro*.

### HMGB1 Facilitated Macrophage Reprogramming towards M1-like Phenotype dependent on PI3Kγ- Erk1/2 pathway

Challenge of ANA-1 with 100 ng/ml rHMGB1, resulted in a transient increase in phosphorylation of PI3Kγ and Erk1/2 within ANA-1, peaking at 30 min, 60 min, respectively (Fig. 3A,B). To furthering confirm the ANA-1 function phenotype reprogramming was PI3Kγ-Erk1/2 dependent following the HMGB1 treatment, AS605240, a PI3Kγ inhibitor and U0126, an Erk1/2 inhibitor were employed, respectively. The ANA-1 was pre-exposure to AS605240 or U0126 and then treated with rHMGB1, the iNOS expression was obviously decreased and the Arg-1 expression down-regulation was rescued (Fig. 3C,D).Taken together, these results demonstrated that HMGB1 facilitating M1 macrophage reprogramming was dependent on PI3Kγ- Erk1/2 pathway.

### Reprogramming towards M1-like Macrophage by HMGB1 promoted Th17 cells expansion

Total CD4^+^T-cells were isolated from spleen of 6 BALB/c mice by positive selection. The purity of CD4^+^T cells was up to 95% by FACS and then co-cultured with macrophages treated by rHMGB1, BSA or without for 4 days. The proportion of Th17 cells increased to 19.21%, which indicated that M1-like macrophage reprogramming by HMGB1 contributed to Th17 cells expansion (Fig. 4A). The culture supernatants were analyzed for IL-17. IL-17 levels were 46.60 ± 6.54 pg/ml, 23.60 ± 5.60 pg/ml and 16.8.60 ± 3.12 pg/ml, (Fig. 4B) among the HMGB1, BSA and control groups, respectively. *p* < 0.001 comparing with BSA and control groups, respectively.

### HMGB1 blockade reduces M1-like macrophages in the heart of EAM

*In vivo*, HMGB1 blockade resulted in a significant reduction in cardiac myocytes necrosis as well as a significant decrease in lymphocyte infiltration and the gross severity scores of untreated and treated samples were significantly different (4.8 ± 0.477 vs. 2.3 ± 0.894, respectively, *p* < 0.001; Fig. 5A). Furthermore, immunofluorescence staining showed that M1-like macrophages infiltration was obviously decreased (3 folds) comparing with EAM (12 folds), *p* < 0.001; Fig. 5B.

## Discussion

As a multifunctional member, macrophages commonly considered to play multiple roles such as providing the first line of defense against pathogens, initiating adaptive immunity by processing and presenting antigens, regulating immune response, mediating inflammation, involvement in autoimmune disease^8^,^15^,^16^, such as collagen-induced arthritis (CIA)^17^, experimental autoimmune encephalomyelitis (EAE)^18^, experimental autoimmune uveitis (EAU)^19^. Furthermore, macrophage functions are settled in response to micro-environmental signals, which drive macrophages reprogramming towards M1 or M2 phenotype. Functional reprogramming of monocyte/macrophage occurs in physiological as well as in pathology milieu, especially the inflammatory factors. Functional phenotype changes of monocyte/macrophage are now considered as a key determinant of disease development and/or regression^20^,^21^,^22^.

In the present work, we demonstrated that HMGB1 could up-regulate iNOS mRNA, protein and activities in macrophages; contributed IL-6, TNF-α, IL-1α, IL-1β and MCP-1 mRNA expression; FCM data furthering showed that HMGB1 increased the proportion of M1-like macrophages (Fig. 2). All these data indicated that HMGB1 facilitated macrophage reprogramming towards a proinflammatory M1-like phenotype *in vitro*. HMGB1, as an important inflammatory factor, binds to the endogenous receptor for advanced glycation endproducts (RAGE)^23^, or exogenous toll like receptor 2/4/9 (TLR2/4/9)^24^,^25^ and CD24/Siglec-10^26^, and induces the expression of proinflammatory cytokines, chemokines, and adhesion molecules^27^; however, HMGB1 ligation with different receptors will have different effects for example, HMGB1 promoted cell proliferation ligation with RAGE; played various biologic activities binding with TLR4^28^. Whether HMGB1 facilitated macrophage reprogramming towards M1-like via TLR4?Therefore, anti-TLR4 mAb was employed. HMGB1 stimulus can’t rescue the proportion of M1-like macrophages following TLR4 blockade (Fig. 4); furthermore, we also demonstrated that PI3Kγ or Erk1/2 inhibition also decreased proportion of M1-like macrophages (Fig. 3); which indicated that HMGB1 facilitate macrophage reprogramming towards M1 functional phenotype was dependent on TLR4-PI3Kγ-Erk1/2 pathway. And the M1-like macrophage promoted Th17 expansion. *In vivo*, infiltrated macrophage was reprogramming towards a proinflammatory M1-like phenotype in EAM; cardiac was protected by monocytes/macrophages depletion or HMGB1 blockade in EAM (Figs 1 and 5); which indicated that HMGB1 may be involve in EAM development partially via promoting macrophage reprogramming.

Our previous data demonstrated that HMGB1 could directly promoted Th17 cells expansion *in vitro*^13^; HMGB1 contributed cardiac fibroblasts/myofibroblasts proliferation, migration, collagen deposition leading the EAM progression^14^; our present data also demonstrated that HMGB1 indirectly contributed Th17 cells expansion by facilitating macrophage reprogramming M1-like phenotype (Fig. 4); and the detailed mechanisms need to be demonstrated for example, M1-like phenotype macrophages contributed to naïve CD4^+^ T cells differentiation into Th17 cells, effector Th17 cells proliferation or anti-apoptosis as well as the signal pathway. Of course, in future, the focus should address on “HMGB1 reprogramming infiltrated monocyte/macrophages or resident macrophages in heart tissue or both”^29^,^30^,^31^. However, our previous and present data at least indicated that HMGB1 truly be involved in EAM development all stages (inflammatory, cardiac myocytes apoptosis, cardiac remodeling); which was mainly dependent on two mechanisms: (1) HMGB1 could promote Th17 cells expansion directly or indirectly by facilitating macrophage reprogramming towards M1-like phenotype; (2) HMGB1 led cardiac fibroblasts/myofibroblasts proliferation, migration, collagen deposition (Fig. 6).

## Conclusion

In conclusion, macrophage reprogramming are now considered as a key determinant of disease development and/or regression. Functional reprogramming of macrophage was associated with pathology milieu, especially the inflammatory factors. In the present study, we clearly demonstrated that HMGB1 facilitated macrophage reprogramming towards M1-like phenotype dependent on TLR4-PI3Kγ-Erk1/2 pathway in EAM development.

## Materials and Methods

### Cells and animals

BALB/c mice were purchased from the Animal Center of Yangzhou University and maintained in Animal Center of Jiangsu University in compliance with the Guide for the Care and Use of Laboratory Animals (NIH Publication No. 85–23, revised 1996). The experimental protocols were approved by the Committee for Ethical Affairs of Jiangsu University (Zhenjiang, China) and the methods were carried out in “accordance” with the approved guidelines. Mice peritoneal macrophages were obtained by peritoneal lavage with 10 ml of RPMI 1640 containing 10% FBS (Gibco, Life Technologies). Cells were incubated 2 h and then washed with PBS to eliminate non-adherent cells. Peritoneal macrophages and ANA-1 macrophages were cultured with RPMI 1640 containing 10% FBS (Gibco, Life Technologies).

### Induction of myocarditis

Mice were inoculated with 100 μg of MyHC-α (MyHC-α_614–629_; Ac-SLKLMATLFSTYASAD-OH), emulsified at a 1:1 ratio in PBS/CFA at days 0 and 7^32^. After 3 weeks, the mice were anaesthetized with pentobarbital sodium (30 mg/g body weight, i.p.), sacrificed by cervical dislocation, and underwent rapid heart excision.

### Macrophage depletion by clodronate-encapsulated liposomes

Dichloromethylene diphosphonate (clodronate, 2.5 g; Sigma) was encapsulated in liposomes formed by a 25:1 w/w ratio of phosphatidylcholine: cholesterol as described^33^. 200 μL clodronate liposome was injected into the mice via caudal vein before the EAM induced and then by 100 μL clodronate liposome/4 days following EAM induced.

### HMGB1 blockade in EAM

The mAb against HMGB1 was produced by hybridoma technology and purified by protein-A affinity chromatography in our lab. For HMGB1 blockade, 100 μg/mouse mAb against HMGB1 (i.p.) was administered every other day according to our lab protocol and the mAb was administered eight times in total.

### Histopathology

Mice hearts were fixed in 10% formalin, paraffin embedded, and stained with hematoxylin and eosin (H&E). Severity scores of myocarditis were graded in double blind manner by two independent investigators according to Dallas criteria, based on the presence of inflammatory cells infiltration and accompanying cardiac myocytes necrosis^34^. The grades were as follows: 0, no inflammatory infiltrates; 1, small foci of inflammatory cells between myocytes; 2, larger foci of greater than 100 inflammatory cells; 3, involving greater than 10% per cross-section; 4, involving greater than 30% per cross-section.

### Immunofluorescence

Immunofluorescence staining of paraffin-embedded mice hearts were performed as described previously^35^. After deparaffinization, rehydration, and antigen unmasking, samples were immersed in blocking buffer for 60 minutes; then PE and FITC labeled antibodies anti-F40/80 and anti-CD11c, (BD Bioscience, USA) were applied overnight at 4 °C. After washing, DAPI added for 10 min. Sections were viewed with a fluorescence microscope (Olympus, Japan) and analyzed using the Image J software.

### NO measurement

ANA-1 macrophages were incubated with recombinant HMGB1 (rHMGB1) (H4652, Sigma Aldrich, USA) (<1 EU/μg endotoxin by LAL test), or without. After 24 h, the supernatant was collected and used for NO detection. NO was measured using Griess Reagent System (Promega, USA), according to the manufacturer’s instructions.

### Quantitative RT-PCR (RT-qPCR)

TNF-α, IL-1α, IL-6, IL-1β, MCP-1, iNOS and Arg-1 message levels were assessed by RT-qPCR as previously described^13^. Briefly, total RNA was isolated from ANA-1 macrophages/Peritoneal macrophages or tissue using TRIzol reagent (Invitrogen Life Technologies, USA) according to the manufacturer’s protocol and reverse transcribed into first-strand cDNA by use of the Moloney murine leukemia virus reverse transcriptase system. After cDNA synthesis, real-time PCR was performed with iQ SYBR Green Supermix (Bio-Rad, USA), using a 7500 Fast Real-Time PCR System (Applied Biosystems, USA) with GADPH or 18s as an internal control. The primers were listed in Table 1. Quantification of gene expression was calculated relative to GADPH or 18s.

### Western blot analysis

Proteins extracted from ANA-1 macrophages were electrophoresed on 12% SDS-PAGE gels and transferred onto polyscreen PVDF transfer membranes (PerkinElmer, USA). Membranes were blocked with 5% (w/v) non-fat dry milk/1% (v/v) Tween 20 in PBS for 2 h at room temperature and incubated overnight with primary antibodies of HMGB1, iNOS, Arg-1, phosphorylated PI3Kγ (p-PI3Kγ), phosphorylated (p-ERK1/2), total ERK1/2 and GADPH or β-actin. After washing, HRP labeled secondary antibodies were added for 1 h at 37 °C temperature. All the antibodies were obtained from Abcam (Abcam, Shanghai, China). Detection was performed with electrochemiluminesce (ECL) and relevant blots quantified by densitometry using the accompanying computerized image analysis program (Amercontrol Biosciences, USA).

### Cytokine assay

Mouse serum was collected and stored at −80 °C until use. IL-6, IL-1β and TNF-α were measured using ELISA kits (Bender MedSystems, Austria), according to manufacturer’s instructions.

### Flow Cytometry Analysis

CD4^+^T cells were isolated by magnetic activated cell sorting (MACS) using CD4 antibodies (Miltenyi Biotec, Germany) according to the manufacturer’s instructions. Isolated T cells were cocultured with macrophages treated by 100 ng/ml rHMGB1 (H4652, Sigma Aldrich, USA), BSA or without, respectively for 4 days^36^. Th17 cell polarization was assessed according previously describe (50 ng/ml PMA and 1 μg/ml ionomycin)^37^ (both from Sigma Aldrich, USA). GolgiPlug (BD Pharmingen, USA) was added during the last 5 h. Cells were fixed and permeabilized and stained with FITC-conjugated anti-IL-17 (BD Pharmingen, USA).

Macrophages were surface-stained with PE-conjugated anti-CD11c and FITC-conjugated anti-F4/80 antibody. After washing with phosphate buffered saline (PBS), stained cells were resuspended and analyzed.

All the samples were analyzed by FACS Calibur (BD Biosciences, USA).

### Macrophage migration assay

Migration assays were performed using 6-well Transwell plates with an 8-μm–pore-size polycarbonate filter (Costar, Cambridge, MA), as previously described^38^. Briefly, ANA-1 were placed in the upper chamber and grown in complete medium. In the lower chamber with or without HMGB1, transwell plates were then incubated for 6 hours at 37 °C in a 5% CO_2_ humidified atmosphere. Migrated macrophages could be readily distinguished from those remaining on the cell surface by their highly refractive morphology. The level of migration was calculated as the percentage of migrated macrophages of the total macrophages within the microscopic field.

### Statistical analysis

All statistical analysis was performed using Graphpad Prism 5 software. Data were expressed as the mean ± standard deviation (SD). Comparisons between groups were performed using the paired t-test or one-way ANOVA with Bonferroni correction. A *p* value of < 0.05 was considered statistically significant.

## Additional Information

**How to cite this article**: Su, Z. *et al.* HMGB1 Facilitated Macrophage Reprogramming towards a Proinflammatory M1-like Phenotype in Experimental Autoimmune Myocarditis Development. *Sci. Rep.* **6**, 21884; doi: 10.1038/srep21884 (2016).

## Supplementary Material

Supplementary Information

## Figures and Tables

**Figure 1:** M1-like macrophage infiltration was increasing and cardiac protection by monocytes/macrophages depletion in EAM. The monocytes/macrophages were deleted by 200 μL clodronate liposome was injected into the mice via caudal vein before the EAM induced and then by 100 μL clodronate liposome/4 days following EAM induced. Heart tissues from C, E, and E-M mice were collected for pathological examination. (**A)** Immunofluorescent staining of infiltrating M1-like macrophages (40×). The cardiac sections taken on day 21 from C and E mice were stained for F4/80^+^ CD11C^+^ macrophages. The proportion of F4/80^+^ CD11C^+^ macrophages was quantified using the Image J software (right panel). (**B)** H&E stained sections (40×). Myocarditis severity scores in the E and E-M group were as follows: E group, grade 5 (n = 3), grade 4 (n = 2); E-M, grade 3 (n = 2), grade 2 (n = 2), grade 1 (n = 1), and in the C group, grade 0 (n = 3), grade 1 (n = 2). (**C)** Serum IL-6, IL-1β and TNF-α levels in E and E-M groups were evaluated by ELISA. *compared with control, ^#^compared with EAM. Data were means ± SD from 5 different mice. *p*-values were calculated using the paired t-test or one-way ANOVA with Bonferroni correction. *p* < 0.05 was considered statistically significant. C, E and E-M represented control, EAM and EAM with monocyte/Mφ depletion group, respectively.

**Figure 2:** HMGB1 promoted macrophage migration and facilitated macrophage polarization *in vitro*. (**A)** iNOS mRNA expression in macrophages. Cells were treated by 50, 100, 250, 500 ng/mL rHMGB1 treatment, LPS as the positive control. Values were expressed compared with 18s. (**B)** iNOS and Arg-1 mRNA expression in ANA-1 macrophages and peritoneal macrophages. Cells were treated with or without the rHMGB1 treatment, LPS as the positive control. Values were expressed compared with 18 s. (**C)** iNOS and Arg-1 protein levels in ANA-1 macrophages. GAPDH was examined as a loading control. (**D)** iNOS activies detection. Data were presented as 540 nm OD values. (**E)** IL-6, TNF-α, IL-1α, IL-1β and MCP-1 mRNA expression. Values were expressed as IL-6, TNF-α, IL-1α, IL-1β and MCP-1 compared with GADPH. (**F)** HMGB1 increased the proportion of CD11c^+^F4/80^+^ macrophages. 100 μg/ml Anti-TLR4 mAb pre-treated one of three groups ANA-1 cells; then cells were cultured with 100 ng/mL rHMGB1 or BSA for 24 h. The markers were measured by FCM. Representative data of three independent experiments was shown. (**G**) Cell migration assay. Cells were performed using 6-well Transwell plates with an 8-μm–pore-size polycarbonate filter, 1 × 10^5^ ANA-1 cells were placed in the upper chamber and grown in complete medium. In the lower chamber with or without rHMGB1, transwell plates were then incubated for 6 hours at 37 °C in a 5% CO_2_ humidified atmosphere. All the data were means ± SD from three independent experiments. *p*-values were calculated using the paired t-test or one-way ANOVA with Bonferroni correction. *p* < 0.05 was considered statistically significant. *NS* means no statistical significance. C, L and H represented control, LPS and HMGB1 group, respectively.

**Figure 3:** HMGB1 Facilitated Macrophage Reprogramming towards M1-like dependent on PI3Kγ- Erk1/2 pathway. (**A,B)** HMGB1 activated the PI3Kγ/Erk1/2 in ANA-1. ANA-1 was treated by 100ng/ml rHMGB1. At the points indicated, cells was harvested; phosphorylated PI3Kγ and Erk1/2 levels were assessed by western blot. Representative blots were shown above and densitometric analyses below. (**C)** iNOS and Arg-1 mRNA expression in HMGB1-treated ANA-1 macrophages with/without AS605240 or U0126 pre-exposure for 1h. Values were expressed as iNOS and Arg-1 compared with 18 s. Data were means ± SD from three independent experiments. *p*-values were calculated using the paired t-test. *p* < 0.05 was considered statistically significant.

**Figure 4:** M1-like macrophages promoted Th17 cells expansion. (**A**) Th17 cells expansion caused by HMGB1 reprogramming macrophages *in vitro*. The macrophages were pre-treated by 100ng/ml rHMGB1, BSA or without for 24 h; after washing, the reprogramming macrophages were co-cultured with total CD4^+^T cells for 4 days. Cells were fixed, followed by permeabilization and intracellular cytokine staining for IL-17. The frequency (%) of IL-17 producing CD4 T-cells gated were shown according to their expression of IL-17. The experiments were repeated three times with similar results. (**B,C**) After a 4-day co-culture of CD4^+^ T cells and macrophages, cells culture supernatants were analyzed for the presence of IL-17. Data were shown as the mean ± SD. *p*-values were calculated using the paired t-test. *p* < 0.05 was considered to be statistically significant. *comparing with control, ^#^comparing with BSA group.

**Figure 5:** HMGB1 blockade reduces M1-like macrophages in the heart of EAM Heart tissues from C, E, and E-B mice were collected for pathological examination. (**A)** H&E stained sections (40×). (**B)** Immunofluorescent staining of infiltrating M1-like macrophages. The cardiac sections taken on day 21 from C, E, and E-M mice were stained for F4/80 ^+^CD11C^+^ macrophages. The proportion of F4/80 ^+^CD11C^+^macrophages was quantified using the Image J software (low panel). Data were means ± SD from 5 different mice. *comparing with E group. *p* < 0.05 was considered statistically significant. (**C,E**) and E-B represented control, EAM and EAM with HMGB1 blockade group, respectively.

**Figure 6:** The possible mechanisms of HMGB1 in EAM development.

**Table 1:** The primers used in the present study.

Genes	Sequence	Size (bp)
IL-6	5′-TGGAGTACCATAGCTACCTGG-3′	188
	5′-AAAAAGTGCCGCTACCCTGA-3′	
TNF-α	5′-GAAAGAAGCCGTGGGTTGGA-3′	268
	5′-ATCCCATGCCTAACTGCCCT-3′	
IL-1α	5′-AAGTCTCCAGGGCAGAGAGG-3′	285
	5′-TGATACTGTCACCCGGCTCT-3′	
IL-1β	5′-CCCTGCAGTGGTTCGAGG-3′	208
	5′-GACAGCCCAGGTCAAAGGTT-3′	
MCP-1	5′-ACTTCGTGGAGGTAGCAACG-3′	222
	5′-TTTGCGGTACCTCTTGGGAC-3′	
iNOS	5′-AACTTGTTTGCAGGCGTCAG-3′	127
	5′-CACATTGCTCAGGGGATGGA-3′	
Arg-1	5′-ACATTGGCTTGCGAGACGTA-3′	109
	5′-ATCACCTTGCCAATCCCCAG-3′	

## References

[b1] GordonS. & MartinezF. O. Alternative activation of macrophages: mechanism and functions. Immunity 32, 593–604, 10.1016/j.immuni.2010.05.007 (2010).20510870

[b2] MotwaniM. P. & GilroyD. W. Macrophage development and polarization in chronic inflammation. Semin Immunol, 10.1016/j.smim.2015.07.002 (2015).26216597

[b3] DesaiB. N. & LeitingerN. Purinergic and calcium signaling in macrophage function and plasticity. Front Immunol 5, 580, 10.3389/fimmu.2014.00580 (2014).25505897PMC4245916

[b4] MillsC. D., ThomasA. C., LenzL. L. & MunderM. Macrophage: SHIP of Immunity. Front Immunol 5, 620, 10.3389/fimmu.2014.00620 (2014).25538705PMC4255611

[b5] MantovaniA. *et al.* The chemokine system in diverse forms of macrophage activation and polarization. Trends Immunol 25, 677–686, 10.1016/j.it.2004.09.015 (2004).15530839

[b6] MosserD. M. & EdwardsJ. P. Exploring the full spectrum of macrophage activation. Nat Rev Immunol 8, 958–969, 10.1038/nri2448 (2008).19029990PMC2724991

[b7] GordonS., PluddemannA. & Martinez EstradaF. Macrophage heterogeneity in tissues: phenotypic diversity and functions. Immunol Rev 262, 36–55, 10.1111/imr.12223 (2014).25319326PMC4231239

[b8] RuckerlD. & AllenJ. E. Macrophage proliferation, provenance, and plasticity in macroparasite infection. Immunol Rev 262, 113–133, 10.1111/imr.12221 (2014).25319331PMC4324133

[b9] AnderssonU. & TraceyK. J. HMGB1 is a therapeutic target for sterile inflammation and infection. Annu Rev Immunol 29, 139–162, 10.1146/annurev-immunol-030409-101323 (2011).21219181PMC4536551

[b10] HarrisH. E., AnderssonU. & PisetskyD. S. HMGB1: a multifunctional alarmin driving autoimmune and inflammatory disease. Nat Rev Rheumatol 8, 195–202, 10.1038/nrrheum.2011.222 (2012).22293756

[b11] MagnaM. & PisetskyD. S. The role of HMGB1 in the pathogenesis of inflammatory and autoimmune diseases. Mol Med 20, 138–146, 10.2119/molmed.2013.00164 (2014).24531836PMC3966993

[b12] LiuY. *et al.* IL-17 contributes to cardiac fibrosis following experimental autoimmune myocarditis by a PKCbeta/Erk1/2/NF-kappaB-dependent signaling pathway. Int Immunol 24, 605–612, 10.1093/intimm/dxs056 (2012).22531062

[b13] SuZ. *et al.* HMGB1 blockade attenuates experimental autoimmune myocarditis and suppresses Th17-cell expansion. Eur J Immunol 41, 3586–3595, 10.1002/eji.201141879 (2011).21928275

[b14] SuZ. *et al.* Up-regulated HMGB1 in EAM directly led to collagen deposition by a PKCbeta/Erk1/2-dependent pathway: cardiac fibroblast/myofibroblast might be another source of HMGB1. J Cell Mol Med 18, 1740–1751, 10.1111/jcmm.12324 (2014).24912759PMC4196650

[b15] HumeD. A. The Many Alternative Faces of Macrophage Activation. Front Immunol 6, 370, 10.3389/fimmu.2015.00370 (2015).26257737PMC4510422

[b16] ZellerI. & SrivastavaS. Macrophage functions in atherosclerosis. Circ Res 115, e83–85, 10.1161/CIRCRESAHA.114.305641 (2014).25477492PMC4414311

[b17] KrauszS. *et al.* Angiopoietin-2 promotes inflammatory activation of human macrophages and is essential for murine experimental arthritis. Am J Cardiovasc Pathol 71, 1402–1410, 10.1136/annrheumdis-2011-200718 (2012).22730375

[b18] van StrienM. E. *et al.* Tissue Transglutaminase contributes to experimental multiple sclerosis pathogenesis and clinical outcome by promoting macrophage migration. Brain Behav Immun, 10.1016/j.bbi.2015.06.023 (2015).26133787

[b19] CoplandD. A. *et al.* Monoclonal antibody-mediated CD200 receptor signaling suppresses macrophage activation and tissue damage in experimental autoimmune uveoretinitis. Am J Pathol 171, 580–588, 10.2353/ajpath.2007.070272 (2007).17600119PMC1934542

[b20] SicaA., ErreniM., AllavenaP. & PortaC. Macrophage polarization in pathology. Cell Mol Life Sci, 10.1007/s00018-015-1995-y (2015).PMC1111354326210152

[b21] WijesunderaK. K. *et al.* M1- and M2-macrophage polarization in thioacetamide (TAA)-induced rat liver lesions; a possible analysis for hepato-pathology. Histol Histopathol 29, 497–511 (2014).2412740010.14670/HH-29.10.497

[b22] SicaA., InvernizziP. & MantovaniA. Macrophage plasticity and polarization in liver homeostasis and pathology. Hepatology 59, 2034–2042, 10.1002/hep.26754 (2014).24115204

[b23] HoriO. *et al.* The receptor for advanced glycation end products (RAGE) is a cellular binding site for amphoterin. Mediation of neurite outgrowth and co-expression of rage and amphoterin in the developing nervous system. J Biol Chem 270, 25752–25761 (1995).759275710.1074/jbc.270.43.25752

[b24] IvanovS. *et al.* A novel role for HMGB1 in TLR9-mediated inflammatory responses to CpG-DNA. Blood 110, 1970–1981, 10.1182/blood-2006-09-044776 (2007).17548579PMC1976374

[b25] ParkJ. S. *et al.* Involvement of toll-like receptors 2 and 4 in cellular activation by high mobility group box 1 protein. J Biol Chem 279, 7370–7377, 10.1074/jbc.M306793200 (2004).14660645

[b26] ChenG. Y., TangJ., ZhengP. & LiuY. CD24 and Siglec-10 selectively repress tissue damage-induced immune responses. Science 323, 1722–1725, 10.1126/science.1168988 (2009).19264983PMC2765686

[b27] DumitriuI. E., BaruahP., ManfrediA. A., BianchiM. E. & Rovere-QueriniP. HMGB1: guiding immunity from within. Trends Immunol 26, 381–387, 10.1016/j.it.2005.04.009 (2005).15978523

[b28] SimsG. P., RoweD. C., RietdijkS. T., HerbstR. & CoyleA. J. HMGB1 and RAGE in inflammation and cancer. Annu Rev Immunol 28, 367–388, 10.1146/annurev.immunol.021908.132603 (2010).20192808

[b29] HulsmansM., SamF. & NahrendorfM. Monocyte and macrophage contributions to cardiac remodeling. J Mol Cell Cardiol, 10.1016/j.yjmcc.2015.11.015 (2015).PMC484655226593722

[b30] PerdigueroE. G. & GeissmannF. The development and maintenance of resident macrophages. Nat Immunol 17, 2–8, 10.1038/ni.3341 (2015).26681456PMC4950995

[b31] OkabeY. & MedzhitovR. Tissue biology perspective on macrophages. Nat Immunol 17, 9–17, 10.1038/ni.3320 (2015).26681457

[b32] ErikssonU. *et al.* Interleukin-6-deficient mice resist development of autoimmune myocarditis associated with impaired upregulation of complement C3. Circulation 107, 320–325 (2003).1253843510.1161/01.cir.0000043802.38699.66

[b33] van RooijenN. & HendrikxE. Liposomes for specific depletion of macrophages from organs and tissues. Methods Mol Biol 605, 189–203, 10.1007/978-1-60327-360-2_13 (2010).20072882

[b34] AretzH. T. *et al.* Myocarditis. A histopathologic definition and classification. Am J Cardiovasc Pathol 1, 3–14 (1987).3455232

[b35] SanadaS. *et al.* IL-33 and ST2 comprise a critical biomechanically induced and cardioprotective signaling system. J Clin Invest 117, 1538–1549, 10.1172/JCI30634 (2007).17492053PMC1865027

[b36] DumitriuI. E. *et al.* Release of high mobility group box 1 by dendritic cells controls T cell activation via the receptor for advanced glycation end products. J Immunol 174, 7506–7515, 174/12/7506 [pii] (2005).1594424910.4049/jimmunol.174.12.7506

[b37] ColantonioL., RecaldeH., SinigagliaF. & D’AmbrosioD. Modulation of chemokine receptor expression and chemotactic responsiveness during differentiation of human naive T cells into Th1 or Th2 cells. Eur J Immunol 32, 1264–1273, 10.1002/1521-4141(200205)32:5 (2002).11981813

[b38] RoviezzoF. *et al.* Human eosinophil chemotaxis and selective *in vivo* recruitment by sphingosine 1-phosphate. Proc Natl Acad Sci 101, 11170–11175, 10.1073/pnas.0401439101 (2004).15254297PMC503758

